# Effect Evaluation of Echocardiography on Right Ventricular Function in Patients after the Recovering from Coronavirus Disease 2019

**DOI:** 10.1155/2022/6161015

**Published:** 2022-07-14

**Authors:** Jianqing Yang, Ping Liu, Mang Zhong, Ting Luo, Guolong Lei, Chunfeng Liao

**Affiliations:** ^1^Department of Ultrasound, Changsha First Hospital, Changsha, 410005 Hunan, China; ^2^Respiratory and Critical Care Center, Changsha First Hospital, Changsha 410005, China; ^3^Department of Cardiovascular Medicine, Changsha First Hospital, Changsha, 410005 Hunan, China

## Abstract

This research was aimed at exploring the changes in right ventricular function in patients after the recovery of coronavirus disease 2019 (COVID-19) under echocardiography and providing a reference for the rehabilitation and treatment of COVID-19 patients. Three echocardiographic follow-up examinations were performed on 40 recovered COVID-19 patients and 40 healthy people. Right ventricular function between patients after COVID-19 rehabilitation and healthy people was compared. The mean values of right ventricular fractional area change (RVFAC), tricuspid annular plane systolic excursion (TAPSE), right ventricular ejection fraction (RVEF), right myocardial performance index (RMPI), and tricuspid annular plane systolic speed (S') were compared between patients after COVID-19 rehabilitation and healthy subjects. The technical parameters of two-dimensional speckle tracking were compared. The results showed that the differences in RVFAC, TAPSE, RVEF, and RMPI between COVID-19 patients and healthy controls were not significant during the three follow-up periods (*P* > 0.05). At the first follow-up, the S' was 12.78 cm/s in COVID-19 patients and 13.18 cm/s in healthy subjects. At the second follow-up, the S' was 11.98 cm/s in COVID-19 patients and 12.77 cm/s in healthy subjects. At the third follow-up, the S' was 12.79 cm/s in COVID-19 patients and 13.12 cm/s in healthy subjects. There was no significant difference between the two groups (*P* > 0.05). In addition, there was no significant difference in right ventricular function between COVID-19 patients and healthy controls, and there was no significant difference in cardiovascular symptoms (*P* > 0.05). In summary, COVID-19 had no substantial effect on right ventricular function and better recovery in patients.

## 1. Introduction

Coronaviruses are the largest known positive strand RNA viruses. It is named coronary or coronavirus under electron microscopy and is a key cause of severe respiratory, intestinal, and systemic infections in various hosts including humans and mammals [1, 2]. Coronavirus disease 2019 (COVID-19) has been afflicting people around the world since December 2019. The disease is highly contagious and devastating, has a huge impact on the lives and safety of people throughout the world, and adversely affects interpersonal communication and economic development [3]. COVID-19 can be divided into mild, usual, severe, and critical types. Mild patients usually have a good prognosis and can be cured without complications after isolation therapy [4, 5]. The main clinical manifestations of COVID-19 are fever, cough, and muscle pain [6]. Some patients may have other symptoms, such as sore throat, runny nose, nausea, vomiting, headache, and diarrhea, and some have decreased or even loss of their ability to smell and taste [7]. Severe clinical symptoms are accompanied by dyspnea, acute respiratory distress syndrome, systemic inflammatory response syndrome, sepsis, coagulopathy, and even death [8, 9]. In recent years, COVID-19 has swept the world and posed a great threat to human health. The number of infections has been increasing.

Patients with COVID-19 not only cause lung lesions and symptoms, but it may also affect other organs, such as the heart, liver, and spleen. Infected patients present to the emergency department with cardiovascular symptoms, and approximately 10% of COVID-19 patients eventually develop cardiac injury [10]. Echocardiography is one of the most commonly used examination methods to assess cardiac structure and function and plays a crucial role in the diagnosis, disease evaluation, and prognosis evaluation of cardiovascular diseases [11, 12]. Echocardiographic parameters can not only estimate the hemodynamic status of patients but also measure the diameter of the pulmonary artery, the size, and the overall motion status of the right ventricle to assess the right ventricular function of patients [13]. Capotosto et al. [14] analyzed the potential role of echocardiography in the current critical period and short and long term of COVID-19 and found that echocardiography has an important role in the assessment of cardiac function in COVID-19. Right ventricular function is usually assessed by changes in right ventricular volume. Due to the asymmetry and complex spatial structure of the right ventricular ventricle, conventional two-dimensional echocardiography is not reliable enough to assess right ventricular function [15]. The acquisition of real-time three-dimensional echocardiography images does not need to rely on specific time and direction, so the volume and function of the right ventricle can be assessed in a real-time, accurate, and reliable manner, with positive application value [16]. Echocardiography is of positive significance in assessing right ventricular function in patients after COVID-19 recovery [17].

Echocardiography was performed on patients after recovering from COVID-19, and the results were compared with healthy people. Echocardiography parameters and indexes of patients after recovering from COVID-19 and healthy people were analyzed. The right ventricular function state of patients after recovering from COVID-19 was explored. The technical parameters of two-dimensional speckle tracking of the two groups were measured, and the prognosis of patients after recovering from COVID-19 was analyzed. It was hoped to provide a reference for the recovery and treatment of patients after recovering from COVID-19.

## 2. Materials and Methods

### 2.1. Subjects

In this research, 80 subjects underwent echocardiographic follow-up examination in health treatment centers and rehabilitation referral hospitals of Hunan Province from March 2020 to March 2022. They were divided into the observation group (40 COVID-19 patients) and the control group (40 healthy people). The male to female ratio was 40 : 40, the mean age was 39.42 ± 5.37 years, and the mean age in the observation group was 39.29 ± 5.14 years. Three echocardiographic follow-up examinations were performed on all study subjects, and echocardiographic parameters were compared between the two groups. This research had been approved by ethics committee of hospital.

The inclusion criteria were as follows: (I) patients with complete medical records and ultrasound images, (II) patients whose ages ranged from 18 to 60 years old, (III) patients without major diseases of vital organs, (IV) patients without hereditary and immune diseases, and (V) patients who were willing to sign the informed consent.

The exclusion criteria were as follows: (I) patients with communication problems, (II) patients with mental disorders, (III) patients who were in pregnancy or lactation, (IV) patients who could not receive regular follow-up examinations, and (V) patients who were unwilling to participate in this experiment.

### 2.2. Methods

Echocardiography was performed on patients during the three follow-up visits at 6, 12, and 18 months after discharge from the hospital for COVID-19. The data were compared with those of the 40 healthy objects. Then, the echocardiographic parameters and right ventricular function of the two groups were analyzed.

### 2.3. Echocardiography Examination

GE E95 echocardiograph was used for echocardiographic examination, and the S5-1 probe was selected with a frequency of 1-5 MHz and a frame rate of 50-70 frames/second. N-terminal fragment brain natriuretic peptides (NT-pro BNP) were analyzed by the I2000 automatic chemiluminescence immunoassay instrument. During ultrasonic image collection and examination, the patient was instructed to lie on the left side and breathe calmly, and the chest lead electrocardiogram was connected. The dynamic image collection was set to 5 cardiac cycles. After the patient's image was stabilized and clear, the conventional ultrasound sections of the heart were collected at the left margin of the sternum, the apex of the heart, and the subxiphoid section. The dynamic images of the second, third, and fourth chamber sections of the apex of the heart and the four-chamber sections dominated by the right ventricle were retained. After the inspection, the relevant Q-Lab was employed for the analysis of the saved images offline. All data were completed by a senior echocardiography physician with extensive experience and collated by two experienced attending physicians.

### 2.4. Image Data Measurement

1. Color Doppler ultrasound diagnosis

The right ventricle endocardium margin was manually delineated from the lateral tricuspid ring along the free wall to the apex of the heart and back down the interventricular septum to the septal tricuspid ring at the end-systolic and end-diastolic stages. The right ventricular end-diastolic area and end-systolic area were recorded, and right ventricular fractional area change (RVFAC) was calculated. The tricuspid annular plane systolic excursion (TAPSE) was measured by the M-type ultrasound in the standard four-chamber section, and the tricuspid annular plane systolic speed (S') was measured by tissue Doppler. The right ventricular ejection fraction (RVEF) was measured by the four-dimensional echocardiography. The right myocardial performance index (RMPI) was measured and calculated as shown in Equation (1), in which RDT presented the equal volume diastolic time of the right ventricle, RST presented the equal volume contraction time of the right ventricle, and RET presented the ejection time of right ventricle.

(1) $$\begin{array}{c} \text{RMPI}=\frac{\left(\text{RDT}+\text{RST}\right)}{\text{RET}}. \end{array}$$

(2) The technical parameters of two-dimensional speckle tracking

Dynamic images of apical four-chamber heart, two-chamber heart, three-chamber heart, and four-chamber heart with the right ventricle as the main four-chamber heart were copied in the digital imaging and communication in medicine (DICOM) format from the GE E95 echocardiography machine. The myocardial motion was tracked and analyzed by using a semiautomated two-dimensional speckle tracking technique. If the tracking was not accurate, the point-and-line adjustment could be implemented manually. The width of the custom “region of interest” included the endocardium, myocardium, and epicardium. Acoustic markers were tracked frame by frame in the customized “region of interest” to analyze the left ventricle overall longitudinal strain (the average of the long axial strain of four-chamber heart, three-chamber heart, and two-chamber heart), the right ventricle overall strain, and free wall strain, all of which were analyzed in four-chamber heart image dominated by the right ventricle. The right ventricle and left ventricle functions were quantitatively evaluated.

The technical parameters of two-dimensional speckle tracking mainly included the left ventricular global longitudinal strain (LVGLS), right ventricular free wall longitudinal strain (RVFLS), left atrial storage (LASr), left atrial vessel function (LASc), left atrial pump function (LASp), right atrial storage (RASr), right atrial vessel function (RASc), and right atrial pump function (RASp).

### 2.5. Observation Indexes

General information, including gender, age, and years of education, was compared between the two groups.

The technical parameters of two-dimensional speckle tracking during three follow-ups were analyzed, including LVGLS, RVFLS, LASr, LASc, LASp, RASr, RASc, and RASp.

Measures of right ventricular function, including RVFAC, TAPSE, RVEF, and RMPI, were analyzed in both groups during three follow-ups.

During the three follow-up periods, S' was analyzed in both groups.

The number of the subjects with cardiovascular symptoms, mainly including palpitations, angina pectoris, vertigo, and hypertension, was analyzed in both groups.

### 2.6. Statistical Methods

SPSS 20.0 was used for data statistics and analysis. Mean ± standard deviation (*x̅*±sd) indicated measurement data, and *t*-test was used. Enumeration data were expressed by percentage (%), and *χ*^2^ test was used. *P* < 0.05 was considered statistically significant.

## 3. Results

### 3.1. Comparison of the General Data

Table 1 shows the comparison of the general data of the objects in the two groups. The male-to-female ratio was 20 : 20 in the control group, and that was 20 : 20 in the observation group. The average age of the control group was 39.78 ± 5.64 years old, and that of the observation group was 39.29 ± 5.14 years old. The years of education in the control group were 12.63 ± 2.72 years, and those in the observation group were 12.77 ± 2.34 years. There was no statistical difference in the general data of the two groups (*P* > 0.05), with comparability.

### 3.2. Comparison of Technical Parameters of Two-Dimensional Speckle Tracking during Three Follow-Ups

Figure 1 shows the comparison of the technical parameters of two-dimensional speckle tracking during follow-up between the two groups. Figures 1(a)–1(h) show LVGLS, RVFLS, LASr, LASc, LASp, RASr, RASc and RASp, respectively. At the first, second, and third follow-ups, there was no statistically significant difference in technical parameters of two-dimensional speckle tracking such as LVGLS, RVFLS, LASr, LASc, LASp, RASr, RASc, and RASp between the two groups (*P* > 0.05).

### 3.3. Comparison of Ventricular Function Index

Figure 2 shows the comparison of RVFAC between the two groups during three follow-ups.  Figure 3 shows the comparison of TAPSE between the two groups during three follow-ups.  Figure 4 shows the comparison of RVEF between the two groups during three follow-ups.  Figure 5 shows the comparison of RMPI between the two groups during three follow-ups. There was not significantly different in RVFAC, TAPSE, RVEF, and RMPI between the two groups (*P* > 0.05). This suggested that right ventricular function was not significantly affected in COVID-19 patients.

### 3.4. Comparison of S' between the Two Groups during Follow-Up

Figure 6 shows the comparison of S' during the three follow-up periods between the two groups. At the first follow-up, S' was 12.78 cm/s in COVID-19 patients and 13.18 cm/s in healthy controls. At the second follow-up, S' was 11.98 cm/s in COVID-19 patients and 12.77 cm/s in healthy controls. At the third follow-up, S' was 12.79 cm/s in COVID-19 patients and 13.12 cm/s in healthy controls. S' was lower in COVID-19 patients compared with healthy controls during the three follow-up periods, but there was no significant difference (*P* > 0.05).

### 3.5. Comparison of the Incidence of Cardiovascular Symptoms

Figure 7 is the comparison of the incidence rate of cardiovascular symptoms between the two groups, in which (a) is palpitation, (b) is angina pectoris, (c) is vertigo, and (d) is hypertension. It can be observed that there were 2 cases of palpitation, 2 cases of angina pectoris, 3 cases of vertigo, and 6 cases of hypertension in the control group. There were 3 cases of palpitation, 1 case of angina pectoris, 4 cases of vertigo, and 7 cases of hypertension in the observation group. The incidence rate of cardiovascular symptoms was 35% in both the control group and the observation group, without statistical difference (*P* > 0.05).

## 4. Discussion

With effective prevention and control measures and people's active cooperation, COVID-19 was gradually brought under control in February 2020. However, COVID-19 still spreads in many countries around the world, posing a serious threat to people's lives and health and a huge burden on the global economy and health [18, 19]. COVID-19 may cause pulmonary fibrosis, which may affect the prognosis of patients [20]. Previous studies by many scholars have demonstrated that lung fibers, as sequelae, seriously affect lung function and the quality of life of patients [21, 22]. Pulmonary fibrosis can cause pulmonary hypertension, which leads to altered right ventricular function and affects the quality of life of patients [23, 24]. Therefore, it is necessary to explore the structural and functional changes of the right heart after recovery.

The right ventricular wall is usually thin, and the pulmonary resistance of the normal right ventricle is quite low, so the normal pressure of the right ventricle is also low [25]. Right ventricular function is usually assessed by the size of the right ventricle and the thickness of the right ventricular wall. Echocardiography has been widely recognized by patients for its advantages of convenience, speed, and low cost [26]. RVFAC and TAPSE are vital indexes that reflect the right ventricular function. RVFAC can reflect the systolic function of the right ventricle as well as the longitudinal and transverse systolic functions of the right ventricular myocardium. TAPSE can reflect the longitudinal contraction of the right ventricle. S' can directly assess the motion of the right ventricular wall. Two-dimensional speckle tracking technology can track the movement trajectory of myocardial tissue with different pixels in the region of interest and calculate the relative change of myocardial length at the end of systole and diastole. It is expressed by the ratio of the difference between myocardial length at the end of systole and diastole. Two-dimensional speckle tracking technology can assess RV dysfunction, with no angle dependence of the measured value and good reproducibility, which has positive application value [27]. Yuchi et al. [28] measured the two-dimensional and Doppler echocardiography indexes of the right heart and the two-dimensional speckle tracking echocardiography indexes, and they found that the morphological indexes of the right heart were evidently increased only in the pulmonary hypertension group, and echocardiography was of great value in the evaluation of cardiac function.

Ishiwata et al. [29] used echocardiography to assess the right ventricular function of patients and analyzed the optimal combination of echocardiographic right ventricular function parameters and found that echocardiographic fractional area change (FAC) and RV longitudinal strain (RVLS) have a good evaluation value. The value of echocardiography in evaluating right ventricular function was investigated, three echocardiographic follow-ups of patients after COVID-19 rehabilitation as well as healthy people were analyzed, and the right ventricular function and prognosis of patients after COVID-19 rehabilitation were explored. The results showed that there was no significant difference in RVFAC, TAPSE, RVEF, RMPI, and S' between the two groups, and there was no significant difference in the incidence of cardiovascular symptoms (*P* > 0.05). It showed that right ventricular function was not significantly affected in COVID-19 patients. The technical parameters of two-dimensional speckle tracking were compared between the two groups. During the three follow-up visits, there were no considerable differences in LVGLS, RVFLS, LASr, LASc, LASp, RASr, RASc, and RASp between both groups (*P* > 0.05).

## 5. Conclusion

According to the follow-up echocardiography in patients after the recovery from COVID-19 and healthy people, the right ventricular function in patients after the recovery from COVID-19 was not remarkably affected. The deficiency of this study is that the sample size is small, which requires further research and verification. In the future, patients after recovering from COVID-19 can be further explored in the left cardiac function state and other functional states of the organism, thus providing theoretical support for the treatment and prognosis of COVID-19.

## Figures and Tables

**Figure 1:** Comparison of technical parameters of two-dimensional speckle tracking during follow-up between the two groups. (a–h) LVGLS, RVFLS, LASr, LASc, LASp, RASr, RASc, and RASp.

**Figure 2:** Comparison of RVFAC between the two groups during three follow-ups.

**Figure 3:** Comparison of TAPSE between two groups during three follow-ups.

**Figure 4:** Comparison of RVEF between the two groups during follow-up.

**Figure 5:** Comparison of RMPI between two groups during three follow-ups.

**Figure 6:** Comparison of S' between the two groups during three follow-ups.

**Figure 7:** Comparison of incidence of cardiovascular symptoms between the two groups: (a) palpitation; (b) angina pectoris; (c) vertigo; (d) hypertension.

**Table 1:** Comparison of general data between the two groups (*x̅*±sd).

	Male/female	Age (years)	Years of education (years)
Control group	20/20	39.78 ± 5.64	12.63 ± 2.72
Observation group	20/20	14 ± 5 ± 39.29	12.77 ± 2.34
*P*	>0.05	>0.05	>0.05

## Data Availability

The data used to support the findings of this study are available from the corresponding author upon request.
